# Comparison of continuous subcutaneous insulin infusion and insulin glargine-based multiple daily insulin aspart injections with preferential adjustment of basal insulin in patients with type 2 diabetes

**DOI:** 10.3892/etm.2014.1866

**Published:** 2014-07-29

**Authors:** GUAN-QI GAO, XUE-YUAN HENG, YUE-LI WANG, WEN-XIA LI, QING-YU DONG, CUI-GE LIANG, WEN-HUA DU, XIAO-MENG LIU

**Affiliations:** 1 Department of Endocrinology, Linyi People’s Hospital, Linyi, Shandong 276003, P.R. China; 2 Department of Clinical Medicine, Linyi People’s Hospital, Linyi, Shandong 276003, P.R. China

**Keywords:** type 2 diabetes, insulin aspart, glargine insulin, hypoglycemia

## Abstract

The purpose of this study was to evaluate and compare multiple daily injection (MDI) therapy of bolus insulin aspart and basal insulin glargine with continuous subcutaneous insulin infusion (CSII) with aspart in patients with type 2 diabetes mellitus (T2DM). It was assessed whether MDI was capable of controlling glycemic index with a higher efficacy than CSII by preferential adjustment of basal insulin with a lower total daily insulin dosage in T2DM. Two hundred patients with T2DM were enrolled in the study and randomly assigned to CSII (n=100) and MDI (n=100; aspart immediately prior to each meal and glargine at bedtime) groups for 12 weeks of therapy. During the last week of each treatment period, the subjects wore a continuous glucose monitoring system for 2–3 days. The dosage of basal insulin was preferentially adjusted to control prior-meal blood glucose levels, and the characteristics of insulin dosage were analyzed. No statistically significant differences were observed between the two groups in hemoglobin A1c (HbA1c), which dropped from 10–11% prior to therapy to 7–7.5% after 12 weeks. After 12 weeks, good glycemic level control was achieved in all patients in the MDI and CSII groups. A statistically significant difference in the dose of insulin between the CSII and MDI groups was observed (P<0.001). In conclusion, no significant differences were found between the two therapies in the incidence of hypoglycemia and HbA1c for the 12 weeks. The basal insulin dosage was significantly decreased in the MDI group compared with that in the CSII group, but the CSII group was superior to MDI group in decreasing fasting blood glucose and shortening the time required for hypoglycemia to meet the targeted level.

## Introduction

Continuous subcutaneous insulin infusion (CSII) therapy with an external pump and multiple daily injection (MDI) therapy are two of the currently selected methods of insulin treatment for diabetes. MDI therapy for diabetes requires bolus injections of rapid or short-acting insulin prior to each meal and a long-acting insulin injection once or twice per day for basal insulin coverage. Control of postprandial glycemia with rapid-acting insulin has been shown to be more effective than that with normal human insulin (1,2). Long-acting insulin, such as insulin glargine, is suitable as a basal insulin therapy in diabetes (3,4). CSII therapy produces a higher efficacy than MDI and improvements in insulin pump technology have resulted in an increase in patient preference (5–10). However, occasionally patients may have to temporarily discontinue CSII therapy due to skin problems, pump malfunction or physical activity. It has been shown that MDI therapy is at least equivalent in its action to CSII (10).

Type 2 diabetes mellitus (T2DM) is characterized by a progressive reduction in β-cell secretion of insulin and mass together with insulin resistance (11). The incidence rate of T2DM has been reported to be 9.7 % in China (12) and Chinese patients with T2DM have shown more significant β-cell deterioration than patients of other genealogies (13). Insulin preparation and medication have undergone rapid progress; however, the amount of insulin injected falls short of what is physiologically secreted in individuals without T2DM. Furthermore, insulin therapy may cause weight increases, hypoglycemia and iatrogenic hyperinsulinemia, which can increase insulin resistance and the potential risks of vascular disease (14). High doses of insulin can induce insulin resistance in diabetic rats, whilst intermediate doses can maximally improve insulin sensitivity (10); therefore, studies investigating the optimal insulin dosage are required. Numerous investigations in patients with type 1 diabetes mellitus (T1DM) have shown that CSII therapy was more efficacious than MDI therapy (15,16), since CSII decreased the dose of insulin required to a greater degree (17–19). Phillip *et al* (20) demonstrated that the higher dose of insulin required with MDI in patients with T1DM, the more marked the insulin decrease subsequent to switching to CSII. Conversely, Monami *et al* (21) showed by meta-analysis of insulin replacement in patients with T2DM that the daily dose of insulin with CSII was not significantly different from that with MDI therapy. Similarly, a study of Indian patients with T2DM showed no significant differences in the total daily dose of insulin when therapy was transitioned from MDI to CSII for six months (22).

The dysfunction of β cells has been found to be a major contributing factor in Chinese patients with T2DM (13); therefore, insulin remains the first choice of therapy. However, as previously discussed, this treatment may result in weight increase, hypoglycemia and iatrogenic hyperinsulinemia, thus increasing the potential risks of insulin resistance, vascular disease and sleep apnea syndrome (14,23–26). Bruttomesso *et al* (15,17) and Hoogma *et al* (27) found that patients with T1DM using CSII required a lower insulin dosage, as compared with those using MDIs. In the present study, it was hypothesized that insulin dosage adjustment may also improve therapy for patients with T2DM. In China, MDI therapy of bolus insulin aspart and basal insulin glargine and CSII are mainly used for glycemic control and treatment of T2DM in hospitalized patients with T2DM. There currently have not been enough relevant investigations demonstrating the optimal insulin dosage in Chinese patients with T2DM. In this study, the insulin dosage characteristics of 200 hospitalized patients with T2DM who were treated with CSII and MDI therapy were investigated.

## Patients and methods

### Subjects

Two hundred patients with T2DM (80 females and 120 males) were recruited for this study. All subjects were hospitalized between January 2011 and July 2013 in the Department of Endocrinology at Linyi People’s Hospital (Linyi, China). The diagnosis of T2DM was established on the basis of the 1999 Diabetes Diagnostic Criteria of the World Health Organization. Subjects hospitalized for insulin treatment due to poor glycemic control and newly diagnosed patients with high blood glucose were enrolled. Subjects prescribed other oral hypoglycemia agents, with the exception of metformin, were excluded and none of the subjects received basal insulin regimen intensification prior the antidiabetic treatment.

Subjects with impaired renal or hepatic function and those who were pregnant or breast-feeding, had malignancies, impaired cardiac function, hypoglycemia unawareness, acute infection or acute complications (such as diabetic nonketotic hyperosmolar coma, diabetic ketoacidosis and diabetic lactic acidosis) were excluded from the study. Investigators and patients were blinded to the therapy sequence up to the point of subject randomization. Subjects were randomly divided into a CSII or MDI group, according to their hospitalization number. One hundred subjects (60 males and 40 females) were randomly assigned to continued therapy with CSII and 100 subjects (60 males and 40 females) to therapy with MDI for 12 weeks. Subjects in the MDI group were administered insulin aspart immediately prior to each meal and then insulin glargine before bed. In the CSII group, all patients received insulin; 32 had peripheral neuropathy, 18 had retinopathy and six had large vessel diseases. In the MDI group, all patients received insulin; 31 subjects had peripheral neuropathy, 18 had retinopathy and seven had large vessel diseases.

### Ethics statement

The investigation was approved by the Medical Ethics Committee of Linyi People’s Hospital. All subjects were patients admitted to the Department of Endocrinology and all patients signed a consent form allowing their information to be stored in the hospital database and used for this study. The consent form was approved by the Medical Ethics Committee of Linyi People’s Hospital.

### Investigation design and method

No oral hypoglycemic drugs, with the exception of metformin, were used during the insulin treatment in the present study. The initial dosage for all subjects was 0.3–0.4 IU/kg/day. The MDI group was treated with insulin aspart (Novo Nordisk, Bagsværd, Denmark) injected subcutaneously prior to each of the three meals in the day, as well as a single basal bedtime injection of insulin glargine (Lantus^®^, Sanofi-Aventis Pharmaceuticals, Mumbai, India) daily, for 12 weeks. The initial glargine-based insulin injections accounted for 60% of the total daily dose and the insulin aspart accounted for 40%. The CSII group was treated with insulin aspart using insulin pumps (Medtronic, Northridge, CA, USA). In the CSII group, the initial basal dose, which accounted for 60% of the total daily amount, was divided into the following four periods of the day: midnight-4:00 a.m., 4:00–9:00 a.m., 9:00 a.m.-9:00 p.m. and 9:00 p.m.-midnight. The three pre-meal doses together accounted for 40% of the total daily dose and were administered for 12 weeks. Blood glucose levels were monitored using a stable blood glucose-monitoring device from LifeScan (Johnson & Johnson Company, Milpitas, CA, USA). Blood glucose levels were measured from finger-stick blood samples eight times per day (before each of the three meals, 2 h later and at 10:00 pm and 3:00 am). The diet of all subjects was regulated according to the China Guideline for T2DM. The basal insulin dose was preferentially adjusted to control the blood glucose when the pre-meal blood glucose level was >9 mmol/l or the postprandial glucose (PBG) was <6 mmol/l according to the features of the PBG state in patients with T2DM (15,26). Pre-meal doses were distributed evenly among the three meals. Basal insulin doses were titrated to target fasting glucose between 4.0 and 7.0 mmol/l. Pre-meal insulin doses were adjusted according to 2-h PBG levels to achieve the target of ≤11.0 mmol/l. If the subject achieved two consecutive days at this level, the length of time required to achieve the target, total daily insulin doses, daily basal insulin doses, blood glucose fluctuations and hypoglycemic episodes were calculated. Hypoglycemic episodes were classified as ‘severe hypoglycemia’ when patients were not able to treat the episode themselves and blood glucose was ≤3.9 mmol/l, ‘symptomatic hypoglycemia’ when patients were able to treat the episode and blood glucose was ≤3.9 mmol/l, and ‘relative hypoglycemia’ when patients exhibited symptoms of hypoglycemia but blood glucose was either >3.9 mmol/l or not measured (28). Hypoglycemic episodes were evaluated as all events (all episodes occurring over a 24-h period) and nocturnal events (episodes occurring between 11:00 p.m. and 6:00 a.m.). Once glycemic control was stabilized for 3 days, the daily insulin dose was calculated when the pre-meal glucose and PBG were <7.01 and 11.09 mmol/l, respectively. The state of hypoglycemia was defined as blood glucose levels ≤3.9 mmol/l or where symptoms of hypoglycemia resolved with administration of oral carbohydrates, and a decrease in basal insulin or regular insulin dose according to pre-meal glucose and PBG.

### Statistical analysis

All statistical data analyses were performed using SPSS version 13. (SPSS, Inc., Chicago, IL, USA). Descriptive data analyses of the qualitative variables were performed with proportions and percentages. Quantitative variables are presented as the mean ± standard deviation. The variables were analyzed with the independent samples t-test between the CSII and MDI groups. A value of P<0.05 was considered to be statistically significant.

## Results

### Clinical data

No statistically significant differences were observed between the CSII and MDI groups in gender, age, hemoglobin A1c (HbA1c), fasting serum C-peptide, body mass index, fasting blood glucose (FBG) or other clinical data (P>0.05) (Table I).

### Insulin doses and incidence of hypoglycemia

Neither the MDI nor the CSII groups had severe hypoglycemic episodes during the treatment duration, and no statistically significant differences were observed in nocturnal hypoglycemic episodes. Good glycemic level control was achieved in the 100 subjects in the MDI group after 6.88±2.31 days. The mean total daily dosage of insulin was 37.12±10.18 IU (0.58±0.17 IU/kg/day), and the total daily basal and bolus doses were 19.35±7.84 and 17.55±3.52 IU (50.80±8.32 and 49.11±8.32% of the total daily dose), respectively. Good glycemic level control was achieved in the 100 subjects in the CSII group after 5.43±2.30 days. The decrease in HbA1c in the two groups was reached earlier in patients in the CSII group compared with those in the MDI group. The mean total daily insulin dose in the CSII group was 31.68±8.88 IU (0.48±0.16 IU/kg/day), and the total daily basal and bolus doses were 22.77±7.65 and 9.78±2.74 IU (69.13±6.99 and 30.87±6.99% of the total daily dose), respectively (Table II). A significant difference in the dose of insulin was observed between the CSII and MDI groups (P<0.001). Insulin requirements decreased 19.12±2.3% after 12 weeks for good glycemic level control in the two groups. Significant differences were found between the two groups in the total dose of insulin and the basal and bolus doses of insulin per day (P<0.001) (Fig. 1 and Table II). The incidence of hypoglycemia was 5.93% in the MDI group and 1.62% in the CSII group (P<0.01) (Table II).

### Treatment efficacy

The mean HbA1c showed a statistically significant decrease during the course of the experiment for the MDI and CSII groups (Table III). In the MDI group, mean HbA1c decreased from 10.79±1.42 to 7.51±1.28%. In the CSII group, mean HbA1c decreased from 10.86±1.36 to 7.11±1.32%. No significant differences were identified between the groups.

The mean FBG levels in the two groups showed statistically significant baseline to end-point decreases, from 8.61±3.12 to 6.76±1.13 mmol/l in the CSII group and from 8.68±3.32 to 6.85±1.26 mmol/l in the MDI group (P<0.005 for both). No statistically significant differences in baseline to end-point FBG level decreases were observed between the two groups (P>0.05) (Table III).

The mean 2-h PBG level decreased significantly from 15.42±4.78 mmol/l at baseline to 9.87±2.63 mmol/l at the end-point in the CSII group and from 15.60±5.71 to 9.95±2.16 mmol/l in the MDI group (P<0.005 for both). No statistically significant differences in baseline to end-point 2-h PBG level decreases were observed between the two groups (P>0.05) (Table III).

### Changes in insulin doses

The total daily insulin dose in the CSII group decreased from 0.48±0.16 to 0.39±0.23 IU/kg/day after 12 weeks (−0.09±0.22 IU/kg/day), and from 0.58±0.17 to 0.47±0.19 IU/kg/day after 12 weeks in the MDI group (−0.11±0.21 IU/kg/day); however, the basal and bolus insulin doses as percentages of the total daily dose remained unchanged at the end of the 12-week period (Table IV).

### Blood glucose levels

Blood glucose levels in the CSII group were lower than those in the MDI group (P>0.05) at each time-point; however, good glycemic control was reached in both groups and no statistical differences were observed in FBG levels, 2 h post-breakfast, 2 h post-lunch or 2 h post-supper blood glucose levels or blood glucose levels at 3:00 a.m. between the two groups (Table V). Blood glucose fluctuations for the CSII group were lower than those for the MDI group (P<0.001) (Table V). Insulin requirements decreased 19.12±2.3% after 12 weeks for good glycemic level control in the two groups.

## Discussion

Blood glucose daily fluctuations contribute to oxidative stress, which can cause long-term complications in patients with diabetes (29). Avoiding glucose fluctuations in patients with diabetes is an emerging challenge (30). The data presented indicate that fluctuations in daily blood glucose were narrower for patients undergoing CSII therapy than for those undergoing MDI therapy. The results were consistent with the theory that basal insulin adjustment using CSII therapy in patients with diabetes provides less variable blood glucose levels than long-acting insulin (31). The variability in blood glucose control appears to be particularly significant with regard to long-acting insulin. However, no difference was detected in daily blood fluctuations between CSII and MDI therapies in a previous study of patients with T2DM (32).

Hypoglycemia is one of the main factors for patients with diabetes requiring insulin to achieve tight glycemic control and a reduced likelihood of complications. No statistically significant differences in nocturnal hypoglycemic episodes and hypoglycemia were detected between the two groups in the present study (P>0.05), suggesting that the safety of the MDI therapy may be comparable to that of CSII therapy in subjects with T2DM.

The data presented in this study showed that, in patients with T2DM treated with insulin therapy for 12 weeks, the total daily dose of insulin in the MDI group was significantly greater than that in the CSII group. The basal dose regulation in the MDI group was not convenient and the mutation variation rates of subcutaneous absorption of bolus insulin aspart and basal insulin glargine were considerably greater in the MDI group than those in the CSII group. Three factors contribute to PBG in diabetes: Increases in glycogen output, FBG and absorption of intestinal glucose. In general, increasing the range of 2 h-PBG depends upon increasing the gastrointestinal glucose absorption and glycogen output. However, gastrointestinal glucose absorption is the same in patients with T2DM and healthy subjects (31) Basal insulin may restrict the glycogen output (33) by decreasing both pre-meal blood glucose and FBG levels and partially restraining postprandial hyperglycemia. Although decreasing PBG may be treated using basal insulin, a lower pre-meal insulin dose is still required as a supplement to control PBG. The pre-meal insulin dose may only restrain the absorption-related increase in glucose and some of the output of glycogen. A lower pre-meal dose may decrease the additive effect of the basal dose, therefore avoiding the requirement for adjustments to be made the basal dose. The study by Suzuki *et al* (33) indicated that an increase in basal insulin dose may be an effective method to control HbA1c and FBG in patients with T2DM and showed the dominance of basal insulin treatment.

Due to the adjustment therapy method used in the present study, the total daily bolus insulin dose of the CSII group was 30.87±6.99%; this contrasted with the total daily bolus dose used in the treatment of Korean patients (64.11±12.10%) (34). In the present study, the mean total daily dose of insulin was 31.68±8.88 IU (0.48±0.11 IU/kg/day) for the 100 patients in the CSII group, while in a study of 46 Indian patients with T2DM the daily insulin dose was 44.0±23.7 IU/day (18). In the present study, the total daily bolus dose (17.55±3.52 IU) of the MDI group subjects comprised 49.11±8.32% of the total daily dose, and the mean total daily dose of insulin was 37.12±10.18 IU/day (0.58±0.17 IU/kg/day); these values were both higher than those of the CSII group subjects. In all subjects, the mean total daily dose of insulin was 34.86±9.76 IU and the dose of insulin per unit body weight was 0.53±0.17 IU/kg/day. The total daily bolus and basal insulin doses were 13.75±5.01 and 21.12±7.91 IU (40.07±11.88 and 59.93±11.88% of total daily dose), respectively. These values differed from those in a previous report where the basal/total daily ratio of insulin was 0.23±0.08 and the mean daily dose of insulin was 38.22±14.92 IU/day (35). From studying 200 patients with T2DM and other related research reports (21,22,34), pre-meal and basal dose proportions have been shown to be associated with the total insulin dose. Pre-meal blood glucose levels can be controlled by preferentially regulating basal insulin, making the required total daily dose of insulin lower.

After 12 weeks of application, MDI-treated patients with T2DM had a higher total insulin dose requirement and hypoglycemia incidence and took longer to achieve the targeted glycemic control compared with the CSII-treated patients. Following CSII treatment in patients with T2DM, decreases in bolus dose and increases in basal insulin dose can form an effective method to achieve good glycemic control with a lower total daily dose. However, where factors exist to prevent the use of therapy with insulin pumps, once daily glargine at bedtime combined with aspart administration at each of the three meals should be an effective alternative.

## Figures and Tables

**Figure 1:** Insulin dose distribution of the MDI and CSII groups. ^*^P<0.05 versus MDI group. MDI, multiple daily injection; CSII, continuous subcutaneous insulin infusion.

**Table I:** Demographic characteristics of the subjects.

	Group	
	
Parameter	MDI	CSII
Male/female (n/n)	60/40	60/40^a^
Newly diagnosed patients (n)	36	36^a^
Duration of diabetes (years)	6.78±5.71	6.89±5.79^a^
Age (years)	51.38±11.73	50.58±12.67^a^
BMI (kg/m^2^)	24.41±3.62	24.89±3.47^a^
HbAlc (%)	10.86±1.36	10.79±1.42^a^
FBG (mmol/l)	7.61±3.12	8.68±3.32^a^
2-h PBG (mmol/l)	15.42±4.78	15.60±5.71^a^
FCP (ng/ml)	0.71±0.44	0.72±0.45^a^

Descriptive data are expressed as the mean ± standard deviation.

a P>0.05 versus MDI group.

HbA1c, hemoglobin A1c; BMI, body mass index; FBG, fasting blood glucose; PBG, postprandial blood glucose; FCP, fasting C-peptide; MDI, multiple daily injection; CSII, continuous subcutaneous insulin infusion.

**Table II:** Comparison of insulin doses upon achievement of good blood glucose control at the start of the 12 weeks of therapy.

Group	n	Rate (IU/kg/day)	Basal insulin dose (%)	Bolus insulin dose (%)	Incidence of hypoglycemia (%)
CSII	100	0.48±0.16^a^	69.13±6.99^a^	30.87±6.99^a^	1.62^b^
MDI	100	0.58±0.17	50.89±8.32	49.11±8.32	5.93

Descriptive data are expressed as the mean ± standard deviation.

a P<0.001 and

b P<0.01 versus MDI group.

CSII, continuous subcutaneous insulin infusion; MDI, multiple daily injection.

**Table III:** Comparison of efficacy between the CSII and MDI groups for 12 weeks.

	Group	
	
Parameter	MDI	CSII
HbAlc		
Baseline (%)	10.79±1.42	10.86±1.36
End-point (%)	7.51±1.28	7.11±1.32^a^
Change (%)	−3.47±1.53	−3.75±1.48
P-value	<0.005	<0.005
FBG		
Baseline (mmol/l)	8.68±3.32	8.61±3.12^a^
End-point (mmol/l)	6.85±1.26	6.76±1.13
Change (mmol/l)	−1.83±2.61	−1.85±2.36
P-value	<0.005	<0.005
2-h PBG		
Baseline (mmol/l)	15.60±5.71	15.42±4.78^a^
End-point (mmol/l)	9.95±2.16	9.87±2.63
Change (mmol/l)	−5.65±4.48	−5.56±4.15
P-value	<0.005	<0.005

Descriptive data are expressed as the mean ± standard deviation.

a P>0.05 versus MDI group.

PBG, postprandial blood glucose; FBG, fasting blood glucose; CSII, continuous subcutaneous insulin infusion; MDI, multiple daily injection.

**Table IV:** Comparison of insulin doses upon achievement of good blood glucose control after 12 weeks.

	Group	
	
Parameter	MDI	CSII
Rate (IU/kg/day)	0.47±0.19	0.39±0.23^a^
Basal insulin dose (%)	50.88±8.42	69.23±6.89^a^
Bolus insulin dose (%)	49.12±8.11	30.77±6.99^a^

Descriptive data are expressed as the mean ± standard deviation.

a P<0.001 versus MDI group.

CSII, continuous subcutaneous insulin infusion; MDI, multiple daily injection.

**Table V:** Comparison of blood glucose levels at different times and blood glucose fluctuations after 12 weeks.

	Group	
	
Parameter	MDI	CSII
Rate (IU/kg/day)	0.47±0.19	0.39±0.23^a^
Basal insulin dose (%)	50.88±8.42	69.23±6.89^a^
Bolus insulin dose (%)	49.12±8.11	30.77±6.99^a^
Blood glucose levels (mmol/l)		
Fasting	6.17±0.71	6.06±0.51
2 h after breakfast	8.96±1.51	8.76±1.11
2 h after lunch	9.23±1.21	9.05±0.91
2 h after supper	8.59±1.19	8.19±0.89
3:00 a.m.	6.26±0.89	6.21±0.61
Blood glucose fluctuation (mmol/l)	0.23±0.06	0.19±0.04^b^

Descriptive data are expressed as the mean ± standard deviation.

a P<0.001 and

b P<0.01 versus MDI group.
